The article "A Cross-Sectional Study on Fall Direction and Lower Limb Loading in Response to a Perturbation on Laterally Inclined Platform" was published in 2023. Journal: Appl Bionics Biomech.

# A Cross-Sectional Study on Fall Direction and Lower Limb Loading in Response to a Perturbation on Laterally Inclined Platform

**DOI:** 10.1155/2023/7385119

**Published:** 2023-10-27

**Authors:** Jaison Jacob Mathunny, Hari Krishnan Srinivasan, Ashok Kumar, Varshini Karthik

**Affiliations:** Department of Biomedical Engineering, SRM Institute of Science and Technology, Kattankulathur, Chennai 603203, Tamil Nadu, India

## Abstract

Perturbation-based balance training (PBT) improves reactive stepping in older adults and people with neurological disorders. Slip-induced falls are a threat to older adults, leading to hip fractures. Fall-prone individuals must be trained to regain balance during a fall in the posterolateral direction. This study aims to analyze the characteristics of the reactive step induced by a laterally inclined platform. This cross-sectional study included 46 healthy participants who performed a “lean and release” backward fall using a platform with two inclined angles on each side. Kinovea software was used to analyze the step width. Reactive steps, characterized by crossover or medial foot placement, are preventive measures against posterolateral falls. The first objective was on the narrowed step width that was subjected to analysis using analysis of variance (ANOVA) and Tukey's post hoc assessment, indicating a tendency toward posterolateral falls. As part of our second objective, the inclined platform resulted in uneven loading between the legs, with a preference for the unloaded leg as the reactive leg (*p* < 0.001), as determined by Fisher's exact test and Cramer's V. These characteristics align closely with those observed in modified constraint-induced movement therapy (mCIMT). The angled platform had a significant effect on selecting the reactive leg, particularly at higher angles (*p* < 0.001). Thus, the study suggested that the device is capable of inducing posterolateral falls and exhibited mCIMT characteristics.

## 1. Introduction

A reactive step is a strategical mechanism a person performs physically to recover balance while falling. Ankle and hip responses can avoid a fall caused by a mild or moderate perturbation. However, a stepping response is inevitable for a large perturbation [1].

Large perturbations are applied to a person in two methods: when they are standing or in motion. Logically, slip and trip occur more in persons who walk or run; however, standing perturbations have been widely used in research for perturbation-based balance training (PBT). Repeated PBT is necessary because it has reduced fall incidents in healthy older adults [2–4] and improved postural stability in the stroke population [5, 6] and people with Parkinson's disease [7, 8]. Repeated PBT improved stability control, and this learned skill was seen to be retained in them for about a year [9].

The article "A Cross-Sectional Study on Fall Direction and Lower Limb Loading in Response to a Perturbation on Laterally Inclined Platform" was published in 2023. Journal: Appl Bionics Biomech.

Balance in a person has been challenged and trained with different techniques/devices that require the patient to be in motion (walk) or motionless (stand). The PBT interventions used with the person in motion are motorized treadmill [10–12], split treadmill [13], and trip and slip walkway [14–16]. While a motorized treadmill perturbs both legs, a split treadmill and slip board perturb a single leg to move the center of mass away from the base of support.

Lean and release test [17–19], lateral waist-pull perturbations [20], and Radboud Falls Simulator (RFS) [5, 6] are devices/techniques that researchers have used to generate a reactive step in persons while they stand still. The lean and release forward fall was used for a forward fall replicating a trip fall, and the lateral waist pull addressed lateral fall, focusing on the crossover step. RFS device is an advanced machine that generates unpredictable perturbation in eight directions. Biodex balance and foam blocks have been used as a motionless intervention with mild perturbation to train ankle and hip stability. Another widely used technique is manually pushing or pulling a fall-prone person, but the push or pull force cannot be quantified, making these techniques hard to prove their effectiveness.

Perturbation-related falls can result in bilateral or split falls, with bilateral falls caused by slips being more common in older adults [21]. A posterolateral bilateral fall has been the primary cause of hip fracture due to a fall that strikes directly on the trochanter [22, 23]. Hence, training a fall that occurs in the posterolateral direction would assist an individual to master the motor skill. With repeated practice till the retention stage, they may be able to execute this skill with fewer cognitive resources [9]. Therefore, it is suggested that a fall-prone individual train on a perturbation technology that can induce a posterolateral fall. As a result, we propose a modified lean and release technique with a laterally inclined platform. The inclined platform could result in an uneven weight loading on the legs, similar to the case of individuals with hemiparetic conditions who mostly avoid using their weak limb to train owing to muscle weakness or significant mobility complications that occurred right after the onset of stroke [24].

Apart from lateral waist pull and lean and forward release fall, to the best of our knowledge, all the devices that generated large perturbations were neither portable nor inexpensive. The RFS device was the only device that induced a posterolateral fall as it produced perturbation in the posterolateral and anterolateral directions. The primary objective of this study is to assess the efficacy of inducing posterolateral falls on a laterally inclined platform. This investigation aims to determine the success rate of prompting posterolateral falls through this platform. Additionally, the secondary objective is to explore whether variations in loading of lower limbs, resulting from participants' positioning on the laterally inclined platform, yield valuable characteristics of their initial stepping.

The article "A Cross-Sectional Study on Fall Direction and Lower Limb Loading in Response to a Perturbation on Laterally Inclined Platform" was published in 2023. Journal: Appl Bionics Biomech.

## 2. Methods

### 2.1. Participants

Forty-six young adults (22 females, 25.2 ± 3.21 years old, 66.6 ± 13.6 kg, 166.7 ± 8.92 cm) participated in this study. The participants were healthy and had no history of fall incidents or injuries. The Institutional Ethics Committee of SRM Medical College Hospital and Research Center approved this study, and all the participants gave informed consent to participate.

### 2.2. Experiment Setup and Protocol

The experimental setup consisted of a custom-made lean and released backward fall technique with a laterally inclined platform for perturbation (Figure 1). The lean and release perturbation method has been widely used in people with strokes [25–27], healthy adults [17], and persons with spinal cord injuries [18, 19]. In this study, a camera (Canon PowerShot SX200 IS) was placed on the posterior side of the participant on a tripod at a height of 25 cm. The video containing the participants' kinematic response (step width) and the leg preferred for a reactive step was analyzed using Kinovea software. The validity and reliability of the Kinovea software in accessing gait kinematics against gold standard motion analysis system [28–30] and the measurement of coordinates and distance of Helen Hayes marker set against gold standard AutoCAD [31] showed excellent intraclass correlation (ICC) values of above 0.9. Kinovea software has also been widely used to analyze parameters recorded in the frontal plane [32–34]. Step width was analyzed to find the location preferred by the participants to place their feet. The abovesaid experimental setup, available at the Human Movement Analysis (HuMA) Lab, SRMIST, KTR, was used for this study.

The customized lean and release backward fall system consisted of a wall-attached load cell that measured the weight the participant exerted on the attached strap exercised by the participant while leaning backward (Figure 1). The strap from the load cell assisted the participants in balancing while leaning backward. The participants wore the harness (fall arrest system) for safety reasons. All the participants leaned backward to initiate the trial, with their feet placed on the marking tape that was adhered to the wooden inclined platform (trials 1–4), as instructed by the investigator. A car seat belt buckle was used to release the strap that secured the participant from falling. A screen placed in front of the participants prevented them from viewing the release of the buckle. Thus, the anticipatory strategies of the participants during the fall were avoided. A few trials were not perturbed to avoid anticipatory moves from the participants. At the time of release, the strap connected to the participant was positioned at the sternum to induce a straight backward fall. This aspect ensured that the direction of the fall was not influenced by any other factor except the efforts made by the participant and the laterally inclined platform angle (which affected the straight backward fall to result in a posterolateral fall). When the participant leaned backward, a laptop connected to the load cell via Arduino Uno displayed information about the weight exerted at the extended strap (customized setup). The releaser made sure to release the buckle when the participant's weight applied on the loadcell was 10%–13% of their weight [19] at 6° and 11° trials, respectively. Monitoring the weight ensured an equal amplitude of perturbation among the participants.

The article "A Cross-Sectional Study on Fall Direction and Lower Limb Loading in Response to a Perturbation on Laterally Inclined Platform" was published in 2023. Journal: Appl Bionics Biomech.

We conducted trials on the lean and release backward fall to avoid the first trial effect and choose the best slope angle for perturbation. We observed that most participants could not recover balance with the laterally inclined platform angled above 11°. Hence, it was decided to have two different laterally inclined angles (6° and 11°) to differentiate the perturbation magnitude.

Each participant executed four trials of backward fall. In trial 1 (6° left), the participants stood on a wooden platform laterally inclined by 6° with the left side of the platform raised on a block of 7 cm in height and the other side on the floor. Trial 2 (6° right) followed the same procedure as trial 1, but the right side was lifted high by 7 cm instead of the left. The height of the platform's left side in the third trial (11° left) and right side in the fourth trial (11° right) was increased to 14 cm, resulting in a lateral slope of 11° (Figure 2). The participants were given verbal descriptions of the lean and release methods, specifically to straightened the knee until the buckle was released. Additionally, participants were told to utilize any leg they preferred for this task. Trials 1–4 did not follow any particular order; the left- or right-side raised trials were interchanged randomly. The participants stood on the wooden platform with a heel distance of 29 cm, with their knees not bent. This stance of the participant tilted them with respect to the lateral slope, with their weight being borne more by the leg that was placed lower in each trial.

The article "A Cross-Sectional Study on Fall Direction and Lower Limb Loading in Response to a Perturbation on Laterally Inclined Platform" was published in 2023. Journal: Appl Bionics Biomech.

### 2.3. Data Analysis

During each of the four trials, reactive stepping was analyzed to determine the leg preference in response to loading induced by the lower-placed leg and the step width. A rectangular box measured 79 cm in length and 91 cm in breadth and a vertical midline dividing it was taped on the floor (Figure 3). The grid option of the Kinovea software was calibrated with these values, so that any steps that fell within the rectangular frame were calculated accurately (Figure 3). Before perturbation, the participant's legs were fixed with markers at the calcaneus, and each heel was 14.5 cm away from the midline. Once a reactive step was made, we subtracted 14.5 cm from the foot that crossed the midline and added 14.5 cm to the foot that did not cross the midline to calculate the step width [32]. For example, as shown in Figure 3, when using the Kinovea software in the SW3 case, the distance from midline to foot placement was calculated to be 12.86 cm, resulting in a step width of 1.64 cm (14.5–12.86 cm). This study did not conduct posterior distance-related measurements because all the research that used lean and release technique, either forward or backward fall, made participants fall anteriorly and posteriorly, respectively. To the best of our knowledge, no study has reported otherwise. Therefore, the study only considered measuring step width reduction related to adduction, indicating the influence of posterolateral fall direction when perturbed on the device studied in this article.

### 2.4. Statistical Analysis

The IBM SPSS Statistics version 23 software was used to analyze the data. A one-way analysis of variance (ANOVA) test was used to analyze the effect of the inclined platform angle on step width. A Tukey's honest significant difference (HSD) post hoc analysis was used to determine the significance level of the reactive step width between the left and right sides for the 6° and 11° inclination platform angle. The frequency of the leg preferred for the initial step of a reactive stepping in trials 1–4 was analyzed using Fisher's exact test and was reported in terms of counts and percentages for these categorical data. The Cramer's V post hoc analysis was used to determine the difference in effect size of the leg preferred between 6° and 11° inclination. The statistical significance, alpha, was set at 0.05.

## 3. Results

All 46 participants could complete all four trials. The participants did not report any discomfort, and none got injured. The primary objective of our analysis was to examine the direction of falls induced by the device, with a particular focus on posterolateral falls. Additionally, we investigated the relationship between step width and the magnitude of perturbations caused by the platform, considering two different incline angles on the right and left sides. We conducted an ANOVA test to assess the impact of the inclined platform's angles on step width. Levene's test was conducted to evaluate the homogeneity of variance, and the results indicated a nonsignificant value of 0.453, indicating that variances were similar across all step width values obtained while performing on various inclined platforms'. Our findings demonstrate significant differences in step width associated with varying platform inclinations (<0.001, as shown in Table 1). The post hoc Tukey's HSD test confirmed that the mean difference in step width between the right and left side for the 6° inclination platform was 10.74 cm and that for the 11° inclination platform was 9.16 cm, with a *p*-value < 0.001.

The article "A Cross-Sectional Study on Fall Direction and Lower Limb Loading in Response to a Perturbation on Laterally Inclined Platform" was published in 2023. Journal: Appl Bionics Biomech.

From the normal stance of 29 cm, the step width was reduced in all the trials, which indicated the tendency of the participant to make a reactive step to negotiate a posterolateral fall.

The box plot (Figure 4) illustrates the placement of the leg landing on the floor in reference to step width. The left leg values were purposely provided with a negative sign to plot on the other side of the “0” value for this box plot. The dotted footprint next to each box plot indicates the foot primarily responsible for the maximum and minimum values in the dataset.

The second objective was to investigate the influence of the inclined platform's characteristics on initial step preference, considering both loaded and unloaded legs. It was observed that the unloaded leg was predominantly preferred for the initial step. As the angle of platform inclination increased from 6° to 11°, the percentage of instances where the unloaded leg was preferred also increased, ranging from 73.9% to 87%.

This outcome, observed during backward laterally inclined perturbation, aligns with the characteristics of modified constraint-induced movement therapy (m-CIMT), where a specific leg can be targeted for a task, such as reactive stepping. The results, as shown in Table 2, show that the angle of the lateral inclined platform significantly influenced leg preference (*p*-value < 0.001).

## 4. Discussion

Fall can occur due to intrinsic or extrinsic factors. Here, we focused on backward falls because approximately out of 81%–98% of hip fracture incidents that occur in a year, 40% are due to slip [35]. Besides, the most concerning injuries are caused by bilateral backward fall, which causes hip and wrist fractures in older adults [14] and people with stroke [36]. PBT has assisted the fall-prone population to reduce falls due to extrinsic factors like obstacles, slips, push, and slopes [37]. Being a laboratory-induced fall intervention in a safe environment, the fall-prone older population can benefit from this repeated perturbation, where research has suggested that the skills acquired during PBT can be retained in them for at least 1 year [38]. Studies have shown that motor skills acquired by an individual undergo various stages, starting with learning, slow, consolidation, automatic, and final retention [9]. Any repeated task can impart the skill to the automatic stage where the skill can be executed with less cognitive resource [9]. Hence, we believe that repeated PBT imitating a realistic posterolateral fall can impart the correct technique to a fall-prone individual to tackle a slip fall, so that they can execute a correct reactive step when an unintentional slip incident occurs.

The article "A Cross-Sectional Study on Fall Direction and Lower Limb Loading in Response to a Perturbation on Laterally Inclined Platform" was published in 2023. Journal: Appl Bionics Biomech.

The hypothesis tested using ANOVA (Table 2) indicates that the location of the leg landing during each perturbation differed depending on the degree of the lateral inclined platform angle with a *p*-value < 0.001. An increase in the slope angle resulted in a reduction in step width. Further, the post hoc analysis of multiple comparisons using Tukey's HSD suggested that the step width generated on the left and right sides with the same degree of inclination was nonsignificant.

More specifically, the step width generated at the left and right sides produced a nonsignificant *p*-value of 0.331 and 0.070 for 6° and 11°, respectively. Hence, the study suggests no difference in the step width within the same slope on the two sides. However, considering the leg that was preferred during each perturbation, left- and right-side slopes were differentiated by giving left leg step width values with an opposite sign to map the box plot (Figure 4) reverse to the right-leg landing. Compared to the initial stance step width of 29 cm, the step width had reduced after perturbation. The reduced step width from the original stance reflects that a reactive step was placed toward the medial side, indicating a posterolateral fall. The step width of a reactive step produced by 6° slope perturbation for both the left and right sides was reduced on their respective sides close to the midline by 8.4 and 4.9 cm, respectively. The results suggested that as the perturbation increased to an 11° incline angle, the participants placed a reactive step similar to a backward crossover step. This characteristic of the step width indicated that the fall was in the posterolateral direction. Bair et al. [39] suggested that crossover steps are challenging for the geriatric population due to interlimb collisions, and there is a need for a minimum of two steps to retain a normal stance. We believe this could have made it challenging for the healthy subjects to balance as the slope increased beyond 11°.

The article "A Cross-Sectional Study on Fall Direction and Lower Limb Loading in Response to a Perturbation on Laterally Inclined Platform" was published in 2023. Journal: Appl Bionics Biomech.

The second objective was to analyze the dissimilar loading on the lower limbs caused by perturbation on a laterally inclined platform. Our results suggest that the angle of the inclined platform affects the preferred leg for a reactive step. The leg located at a height on the laterally inclined platform was mainly influenced to act as the reactive leg. The left leg raised at 6° and 11° slopes produced a left leg reactive step of 74% and 87% (Table 2), respectively. Similarly, on the right side, an elevation with a slope of 6° and 11° resulted in a reactive step caused by the right leg with 85% and 94%, respectively. Thus, the study suggests that the laterally inclined angle of the platform can target and influence the leg that needs to act as a reactive leg, while the other leg acts as a supporting leg.

As an extension of this objective, the influence of the preferred leg was correlated with the increased inclination angle of the platform. The 6° inclined platform showed a Cramer's V value of 0.590, with an increase in effect size (0.806) when the inclination angle was increased to 11°. The lateral leaning of the body due to the inclination of the platform has caused an increase in ipsilateral leg loading [40]. Hence, the leg positioned at a height was loaded less, and more weight was borne by the leg placed at a lower level. In this case, the base of support (center of mass) moves to the lower leg. Therefore, the study, conducted with healthy participants, suggests that the possibility of targeting a lower-loaded limb as a reactive leg may depend on the inclination angle of the perturbation platform. This observation raises the potential that in fall-prone individuals, the likelihood of using the lower-loaded leg as the reactive stepping leg could be higher, depending on their individual conditions. We understand that further research in this direction is warranted to validate these hypotheses with the fall-prone populations, and we encourage future investigations to explore this area more comprehensively. The inclination angle may play a significant role in determining the effectiveness of this approach. The results exhibited characteristics resembling those found in mCIMT, which promotes the use of weaker limbs by partially restricting the healthy leg. The mCIMT has been widely used for the lower limb because of the bipedal nature that humans possess [36, 41–44]. Like conventional CIMT, completely restricting the two lower limbs will not work in PBT because both lower limbs have a crucial role in balancing after a perturbation. Research that has used mCIMT interventions has shown improvement in hemiplegic gait parameters [45], balance, and motor functions [46].

The article "A Cross-Sectional Study on Fall Direction and Lower Limb Loading in Response to a Perturbation on Laterally Inclined Platform" was published in 2023. Journal: Appl Bionics Biomech.

The limitation of the study is that the participants used for the study were normal, healthy subjects. Characteristics of a reactive step may change when trials are conducted with subjects with neurological disorders or the geriatric population. Further research involving a broad spectrum of samples of various groups of participants is required to extend these findings into practical design inputs and personalize this portable perturbation device to determine the best-inclined angle of the platform that suits each group. Another limitation is that, as suggested by other studies, mCIMT has improved balance and motor function in people with hemiparetic conditions, but the use of mCIMT in older adults is an unexplored area.

The intervention studied in this work suggests the need to train fall-prone individuals with a PBT that follows a posterolateral fall, as previous research suggested that most hip fractures occur due to the fall in this direction. A laterally inclined platform was used to induce the posterolateral fall, and the step width pattern of the participants suggests the same. The leg placed lower on the laterally inclined platform acted as the restricted limb, whereas the other higher-placed one served as the reactive limb. This output reflects the mCIMT property in this intervention and is believed to be useful in subjects with hemiparetic conditions. It may be helpful to investigate the features of reactive stepping due to reduced base support caused by platform inclination. These factors have increased instability in participants, and analyzing their importance could help create more effective strategies to prevent falls.

## Figures and Tables

**Figure 1:** The whole setup of lean and release backward fall with a laterally inclined platform.

**Figure 2:** Laterally inclined platform setup.

**Figure 3:** Measurement of step width using Kinovea software. (a) The grid in Kinovea software is calibrated to ensure accurate measurements. (b) Step width (SW) measurement: Real Kinovea data are collected, as illustrated in the SW3 of diagram (c). The measured step width is 1.64 cm, which is calculated by subtracting the resultant 12.86 cm from the initial 14.5 cm since the right leg has crossed the midline. Reference distance test: A reference distance test is performed in the background, where a 16.89 cm Kinovea measured distance is validated between stickers placed within a grid section that measures physically 17 cm. (c) SW1 case: SW1 represents a case where the right leg did not cross the midline and is positioned 14.5 cm away from the midline. Therefore, SW1 is 29 cm. SW2 case: SW2 represents a case where the step width is on the midline, resulting in a step width (SW2) of 14.5 cm.

The article "A Cross-Sectional Study on Fall Direction and Lower Limb Loading in Response to a Perturbation on Laterally Inclined Platform" was published in 2023. Journal: Appl Bionics Biomech.

**Figure 4:** The box plot shows the exact width of where each step was placed. The rectangular box in the bottom left corner shows the mean distance from the center of the stance.

**Table 1:** The influence of step width on different inclined platform angles and the comparison between both sides of the leg.

Inclined platform angle	ANOVA test		Tukey's HSD	
	Step width mean (cm)	*p*-value	Mean difference	*p*-value
6° left (left leg raised)	19.42	<0.001	10.74	<0.001
11° left (left leg raised)	8.69			
6° right (right leg raised)	22.90		9.16	<0.001
11° right (right leg raised)	13.73			

**Table 2:** Effect of inclined platform angles on initial leg stepping preference.

Inclined platform angle	Leg dynamics in terms of loading		Initial leg stepping preference		Fisher's exact test (*p*-value)	Phi/Cramer's V (*p*-value)
	Left	Right	Left (%)	Right (%)		
6° left (left leg raised)	Unloaded	Loaded	34 (73.9)	12 (26.1)	<0.001	0.590 (<0.001)
6° right (right leg raised)	Loaded	Unloaded	7 (15.2)	39 (84.8)		
11° left (left leg raised)	Unloaded	Loaded	40 (87)	6 (13)	<0.001	0.806 (<0.001)
11° right (right leg raised)	Loaded	Unloaded	03 (6.5)	43 (93.5)		

## Data Availability

The data that support the findings of this study are available upon request. We are committed to making our data accessible and reproducible, and we encourage interested researchers to contact us for more information.
